# Scientific Evidence of Traditional Chinese Exercise (Qigong) for Chronic Obstructive Pulmonary Disease: An Overview of Systematic Reviews and Meta-Analyses

**DOI:** 10.1155/2022/7728973

**Published:** 2022-08-02

**Authors:** Hongshuo Shi, Ting Liu, Chengda Dong, Kun Zhen, Yuxuan Wang, Pengjun Liu, Guomin Si, Lei Wang, Min Wang

**Affiliations:** ^1^Shandong University of Traditional Chinese Medicine, Jinan, China; ^2^Shandong Provincial Hospital Affiliated to Shandong First Medical University, Jinan, China; ^3^The Second Affiliated Hospital of Shandong University of Traditional Chinese Medicine, Jinan, China

## Abstract

**Background:**

As a traditional Chinese exercise, Qigong has potential benefits for the management of chronic obstructive pulmonary disease (COPD). This overview is aimed at assessing the existing evidence for the intervention of Qigong in COPD so as to provide scientific guidance for clinical decision-making.

**Methods:**

The systematic reviews (SRs)/meta-analyses (MAs) of Qigong for the treatment of COPD were obtained from 7 electronic databases with the search date set at April 5, 2022. Two researchers independently assessed the methodological quality, reporting quality, and evidence quality for the included SRs/MAs using the following tools: the Assessment of Multiple Systematic Reviews 2 (AMSTAR-2), the Preferred Reporting Items for Systematic Reviews and Meta-Analyses 2020 (PRISMA 2020), and the Grading of Recommendations Assessment, Development, and Evaluation (GRADE) system.

**Results:**

A total of 13 SRs/MAs were included in this overview. All SRs/MAs assessed by AMSTAR-2 had more than one critical defect, so all SR/MAs were rated very low. Regarding the assessment of reporting quality, the results of PRISMA 2020 showed that none of the SRs/MAs were fully reported. In addition, the results of the GRADE assessment of the quality of evidence indicated that only 3 outcomes were rated as high quality across all SRs/MAs.

**Conclusion:**

Current evidence suggests that Qigong is effective and safe for the management of patients with COPD. However, the high risk of bias in the original clinical studies and the low quality of the SRs/MAs reduced the reliability of the results.

## 1. Introduction

Chronic obstructive pulmonary disease (COPD) is characterized by persistent airflow limitation, recurrent respiratory symptoms, and extrapulmonary manifestations [1, 2]. According to the World Health Organization, COPD is projected to become the third leading cause of death globally by 2030 [3]. In addition, COPD-related mortality is expected to increase gradually due to increased environmental exposures (smoking, ambient particulate matter, etc.) and an aging population [4]. By 2060, more than 5.4 million people could die each year from COPD and related diseases [1]. Therefore, COPD is an important challenge for global public health. In addition to this, COPD also imposes a huge financial burden on individuals and society as it is associated with high disability rates [5].

Standardized rehabilitation can delay the acute exacerbation and progression of COPD patients and improve their quality of life. Therefore, pulmonary rehabilitation in COPD patients is valued by clinicians and researchers [6]. Exercise is seen as the key to pulmonary rehabilitation, with the main aim of improving aerobic capacity in COPD patients [7]. Qigong, as one of the four pillars of traditional Chinese medicine [8], was rejuvenated in the 1950s to include a series of techniques aimed at improving the physical, mental, emotional, and respiratory health. Since the 1980s and especially the 2000s, there has been considerable interest in Qigong as a potential therapeutic modality [9]. As a mind-body exercise, Qigong incorporates the elements of physical movement, spiritual guidance, and breath control [10, 11], and there are various forms of Qigong, such as Wuqinxi, Baduanjin, Yijinjing, and Liuzijue.

Over the past 5 years, a large number of systematic reviews (SRs)/meta-analyses (MAs) have been completed to assess the potential benefits of Qigong for the health management of patients with COPD. Based on evidence-based medicine theory, SRs/MAs are considered the gold standard for evaluating the benefits of clinical interventions [12]. The overview is a new approach to integrating multiple SR/MAs by evaluating their quality and outcomes, which can provide comprehensive evidence for clinical decision-making and identify critical gaps in evidence use. Therefore, the aim of our study was to critically evaluate the quality of SR/MA related to the effect of Qigong in patients with COPD through a systematic overview.

## 2. Materials and Methods

This research was conducted according to the Cochrane Handbook, and we followed the methods of Huang et al. [13] and Shi et al. [14].

### 2.1. Eligibility Criteria

Eligible studies meet the following criteria: (1) study of research: SRs/MAs of randomized controlled trials (RCTs) reported the efficacy or safety of Qigong in COPD; (2) inclusion of the population: patients identified as having COPD based on diagnostic criteria regardless of their age, nationality, or gender; (3) interventions: the intervention methods for the control group included conventional medicine (CM), routine activities (RA), breathing training (BT), and health education (HE); (4) outcomes: the forced expiratory volume in one second (FEV1), forced vital capacity (FVC), 6-min walking distance (6-MWD), the amount of air exhaled in the first second divided by all of the air exhaled during a maximal exhalation (FEV1/FVC), St George's respiratory questionnaire (SGRQ), COPD assessment test (CAT), percentage of the forced expiratory volume in one second (FEV1%), quality of life (QOL), the World Health Organization on quality of life brief scale (WHOQOL-BREF), medical research council dyspnea scale (MRC), and the percentage of predicted values of FEV1 (FEV1%pred).

Studies that met the following criteria were excluded: (1) network meta-analyses, SRs/MAs without quantitative synthesis, conference abstracts, reviews, editorials, case reports, and replication studies; (2) animal experiments; and (3) the control group used other traditional Chinese exercises.

### 2.2. Search Strategy

Two researchers (YX-W and HS-S) independently searched PubMed, Embase, Cochrane Library, CBM, CNKI, Wanfang database, and VIP database, and the search time ranged from the database establishment to April 5, 2022. A combined search strategy that incorporates keyword search and free-word search was adopted, where the keywords include “Qigong”, “Chronic obstructive pulmonary disease”, “meta-analysis”, and “systematic review”. The search strategy was adjusted to fit different databases. In addition, we manually searched for relevant references to ensure the completeness of the search. We also searched Web of Science and Scopus databases from the database establishment to June 22, 2022. The search strategy for PubMed is shown in Table 1.

### 2.3. Literature Screening and Data Extraction

Two independent researchers (PJ-L and HS-S) conducted the screening of the literature. The retrieved publications were imported into a literature management system (EndNote X9), and the initial screening was performed by firstly removing duplicates and subsequently reading the titles and abstracts. Finally, the full text was read to identify the final literature for inclusion. To ensure data integrity and consistency, the two researchers (K-Z and HS-S) used a predesigned data extraction table to extract the data. The extracts included first author, year of publication, country, number of RCTs (number of subjects), interventions, risk of bias assessment methods, interventions, and main findings.

### 2.4. Quality Evaluation for Inclusion in SRs/MAs

Two independent researchers (YX-W and HS-S) assessed the methodological quality, reporting quality, and evidence quality of the included SRs/MAs. Any disagreements were referred to a third investigator (M-W) for consultation.

#### 2.4.1. Methodological Quality Evaluation

The methodological quality of the included SRs/MAs was assessed using the Assessment of Multiple Systematic Reviews 2 (AMSTAR-2) [15]. The tool contains seven key items (2, 4, 7, 9, 11, 13, and 15). Each item was categorized as “no,” “partially yes,” or “yes” depending on their compliance with the criteria. The overall methodological quality was classified into four levels: high, medium, low, or very low.

#### 2.4.2. Report Quality Evaluation

The Preferred Reporting Items for Systematic Reviews and Meta-Analyses 2020 (PRISMA 2020) [16] was used to assess the quality of the report, and it covers 27 items. Each item can be assessed as “yes,” “partially yes,” or “no,” with a ratio based on the assessment of each item.

#### 2.4.3. Evidence Quality Evaluation

The Grading of Recommendations Assessment, Development, and Evaluation (GRADE) [17] system was applied to assess the quality of evidence for inclusion in the SR/MA outcome indicators. Evidence quality may be downgraded due to the following 5 criteria: risk of bias, inconsistency, indirectness, imprecision, and publication bias. The quality of evidence was categorized as high, moderate, low, and very low.

## 3. Results

### 3.1. Literature Selection

Nine electronic database searches identified 193 publications, 119 of which were excluded after removing duplicates. Afterwards, 13 publications were excluded by screening the titles and abstracts. Then, further screening was performed by reading the full text, and three papers [18–20] were excluded in this step due to their failure to meet the intervention criteria. Ultimately, a total of 13 papers [21–33] were included. The flow chart of literature screening in this study is shown in Figure 1.

### 3.2. Characteristics of the SRs/MAs

The characteristics of the 13 SRs/MAs used for qualitative analysis in this overview are summarized in Table 2. All SRs/MAs were published between 2015 and 2021, with 12 (12/13, 92.3%) [21–28, 30–33] of them published within the last 5 years. In the original study of SRs/MAs included in this overview, the first RCT of Qigong intervention in COPD was published in 2008 by Chen et. al [34]. All included SRs/MAs were published by Chinese scholars, five [21, 22, 27, 28, 31] of which were written in English and eight [23–26, 29, 30, 32, 33] in Chinese. The number of RCTs included per SR/MA ranged from 8 to 30, and the participants in these RCTs ranged from 534 to 3,045. In terms of intervention modality, the control group was treated by CM, RA, BT, and HE, while the experimental group was treated by various types of Qigong or Qigong in combination with the treatments received by the control group. The various types of Qigong included Baduanjin, Liuzijue, Wuqinxi, and Yijinjing. Twelve [21, 23–33] SRs/MAs used the Cochrane criteria for risk of bias assessment of included RCTs, and the remaining 1 SR/MA [22] used the physical therapy evidence database scale. In addition to this, all SRs/MAs were subjected to meta-analysis and all reported positive results.

### 3.3. Quality Assessment

#### 3.3.1. Methodological Quality Assessment

AMSTAR-2 was used to evaluate the methodological quality of the SRs/MAs included in this study, the details of which are given in Table 3. The methodological quality of all SRs/MAs was very low due to multiple deficiencies in critical and noncritical items. The deficiencies in the inclusion of SRs/MAs assessed by AMSTAR-2 were as follows: Item 2 (only 2 [27, 28] SRs/MAs have registered study protocols), Item 7 (none of the SR/MA provided a list of excluded articles), Item 10 (none of the SR/MAs provided a list of funding for RCTs), and Item 15 [21–23, 25, 26, 28] (only 6 SRs/MAs completed the publication bias assessment).

#### 3.3.2. Report Quality Assessment

Detailed information on the quality of the report is presented in Table 4. Although the titles, abstracts, introductions, and discussions of the SRs/MAs included in this overview were reported in their entirety, some reporting deficiencies were still identified in other sections. In Materials and Methods, Item 7 (search strategy), Item 13(e) and (f) (synthesis methods), Item 14 (reporting bias assessment), and Item 15 (certainty assessment) have less than 50% response rate. In the results section, less than half of Item 20(d) (results of syntheses), Item 21 (reporting biases), and Item 22 (certainty of evidence) were reported. Only 2 [27, 28] (2/13, 15.38%) SRs/MAs provided information on the registration of study protocols, which made the quality assessment of Item 24 (registration and protocol) reporting unsatisfactory. In addition to this, only 5 [21, 22, 27, 28, 31] (5/13, 38.46%) SRs/MAs reported conflicts of interest, which rendered Item 26 (competing interests) reporting insufficient.

#### 3.3.3. Evidence Quality Assessment

The 13 SRs/MAs included in this overview contain 73 outcomes. Results of the quality of evidence assessment showed that 3 items were rated as high quality, 17 items were rated as moderate quality, 23 items were rated as low quality, and the remaining 30 items were rated as very low quality. Among the downgrading factors, publication bias (*n* = 58) was the most common downgrading factor, followed by inconsistency (*n* = 52), risk of bias (*n* = 25), imprecision (*n* = 21), and indirectness (*n* = 0). Detailed information on the quality of the evidence is presented in Table 5.

### 3.4. Summary of the Outcomes of the Qigong Intervention COPD

We presented a summary and narrative description of the outcome indicators quantitatively assessed by the SRs/MAs in this overview. Complete information is presented in Table 6.

#### 3.4.1. Effect of Qigong on Exercise Endurance

Twelve SRs/MAs [21, 22, 24–33] reported the effect of Qigong on 6-WMD, and the results indicated that Qigong could significantly improve 6-WMD in COPD patients.

#### 3.4.2. Effect of Qigong on Lung Function

Twelve SRs/MAs [21–31, 33] reported that Qigong could significantly improve FEV1 in COPD patients. Eleven SRs/MAs [22–31, 33] reported the effect of Qigong on FEV1%, of which 10 SRs/MAs [22–31] showed that Qigong could significantly improve FEV1% in COPD patients. Ten SRs/MAs [21–28, 31, 33] reported the effect of Qigong on FEV1/FVC, and the results of 9 SRs/MAs [21–28, 31, 33] indicated that Qigong could significantly improve FEV1/FVC in COPD patients. Six SRs/MAs [21–26] reported that Qigong could significantly improve FVC in COPD patients. In addition, 3 SRs/MAs [25, 27, 33] reported that Qigong could significantly improve FEV1/pred% in COPD patients.

#### 3.4.3. Effect of Qigong on Dyspnea

Three SRs/MAs [25, 28, 30] reported that Qigong could significantly improve MRC in COPD patients.

#### 3.4.4. Effect of Qigong on Quality of Life

Seven SRs/MAs [21, 23, 26, 27, 30–32] reported the effect of Qigong on CAT, and the results of 6 SRs/MAs [21, 23, 27, 30–32] indicated that Qigong could significantly reduce CAT in COPD patients. Three SRs/MAs [21, 26, 27] reported that Qigong could significantly reduce SGRQ in COPD patients. One SR/MA [26] reported that Qigong could significantly improve WHOQOL-BREF in COPD patients. In addition, two SRs/MAs [22, 28] reported that Qigong could significantly improve the quality of life of COPD patients by comprehensively evaluating the effect of Qigong on CAT and SGRQ.

### 3.5. Adverse Events

None of the SRs/MAs quantified the adverse events of Qigong in patients with COPD, and two SRs/MAs [27, 30] descriptively set forth the safety of Qigong in patients with COPD.

## 4. Discussion

COPD rehabilitation is a key approach to COPD treatment recommended by current guidelines, and the recommended approach to rehabilitation includes physical exercise [35, 36]. As an important supplement to the physical exercise of COPD patients, Qigong can achieve the purpose of unity of body and mind through specific movements, breathing techniques, and meditation, thereby regulating the patient's energy (qi) and benefiting the patient's physical, mental, and spiritual health [37]. Although the number of published SRs/MAs on the Qigong treatment for COPD is on the increase, no published overview has so far put them together and assessed their quality. Therefore, an overview of this topic is necessary.

This overview is the first evaluation of Qigong for COPD-related SRs/MAs using AMSTAR-2, PRISMA 2020, and GRADE. More than 90% (12/13, 92.3%) of these SRs/MAs were published in the last five years, indicating the growing interest in Qigong for COPD. However, the quality of the included SRs/MAs was not satisfactory.

### 4.1. Questions about the Quality of the Current Evidence and Recommendations

Based on the details of the AMSTAR-2 assessment, the major factors for the low methodological quality of the included SRs/MAs were as follows: Item 2 (protocol registration, 2/13, 15.38%), Item 7 (exclusion list, 0/13, 0%), Item 10 (funding sources, 0/13, 0%), and Item 15 (publication bias assessment, 6/13, 46.15%). Study protocol registration is important when researchers identify topics for SRs/MAs, which helps improve processing transparency and minimizes selective reporting bias [38]. A list of excluded literature was not provided for all included SR/MAs, which may affect the reproducibility of results and undermine the transparency of the study, making it difficult to ensure the reliability of the results. None of the SRs/MAs provided funding resources, which may increase bias in the reporting of clinical trials, as the results of commercially funded studies may be biased toward the institution in question. In addition, only 6 SRs/MAs were assessed for publication bias, which may lead to less confidence in the results of SRs/MAs.

Regarding reporting quality, the results of PRISMA 2020 showed that, like AMSTAR-2, the study protocol, RCTs funding, and publication bias were not fully reported. In addition, the lack of a complete search strategy, sensitivity analysis, and certainty of evidence assessment are also important reasons for the low quality of the report. Only 2 (2/13, 15.38%) SRs/MAs provided a complete search strategy for all electronic databases, which makes the studies nonreproducible and may also lead to publication bias. Only 5 (5/13, 38.46%) SRs/MAs were subjected to sensitivity analysis, and the absence of sensitivity analysis was detrimental to the stability of the judgmental effect size assessment, resulting in a decrease in the credibility of the results. In addition, none of the SR/MAs reported certainty of evidence, which is significant for our study.

For the assessment of evidence quality, only 3 of the 73 outcomes assessed were rated as high quality. A closer analysis revealed that publication bias (58/73, 79.45%) and inconsistency (30/73, 71.23%) were the main factors contributing to the downgrading of the quality of the evidence. Publication bias arises due to insufficient assessment of publication bias and an insufficient number of RCTs with relevant outcomes. Further analysis revealed a high degree of heterogeneity in many of the results, likely due to clinical and methodological differences in the included RCTs. Since the included RCTs include COPD patients of different ages, genders, and clinical stages, there is no uniform standard regarding the intervention time, frequency of intervention, and movements of Qigong. Due to the adoption of different measurement tools and methods, the same outcome measures may also differ in different studies, which is also a potential cause of heterogeneity.

Through a narrative overview of the outcome indicators of COPD treated with Qigong, we found that Qigong is effective and safe for COPD patients. Qigong has significant effects on improving lung function, exercise tolerance, dyspnea, and quality of life in COPD patients. However, caution is still required when recommending Qigong for COPD treatment, as the included SRs/MAs are of low quality and may not serve as a scientific basis for clinical practice by clinicians.

Our study suggests that Qigong may be a promising complementary therapy for COPD, but due to the overall low quality of the included evidence, the following is strongly recommended for the carrying out of SRs/MAs and RCTs in the future. For TCM-related SRs/MAs, registration on international platforms (e.g., Cochrane Library, PROSPERO, INPLASY, and JBI) and/or early publication of protocols are highly recommended. When conducting SRs/MAs, researchers should provide a complete list of search strategies for each electronic database, a list of excluded literatures, and the source of funding for the RCT to increase the transparency and reduce the publication bias of the article. To improve the reliability of the results, publication bias assessment and sensitivity analysis should be performed.

### 4.2. Implications for Future Practice and Research

The improvement in exercise capacity, lung function, and quality of life in COPD patients may be related to the exercise pattern of Qigong, which, as a light to moderate aerobic exercise, is well suited for COPD patients with low exercise tolerance [39]. Qigong includes musculoskeletal stretching, breathing regulation, and mental coordination. These motor components may be the key to enhancing lung function and diaphragm capacity in COPD patients. In addition, Qigong also involves mental focus and relaxation, which can increase the sense of well-being in COPD patients, thus promoting the patients' mental health and increasing compliance with Qigong exercises.

A prerequisite for high-quality SRs/MAs is that the original studies included are of high quality. Clinical researchers should improve the top-level design of clinical trials through comprehensive evaluation and sophisticated analysis. Notably, Consolidated Standards of Reporting Trials (CONSORT) should be used to improve the quality of evidence from RCTs [40]. Careful design, rigorous implementation, and complete reporting of RCTs are considered gold standards for avoiding the research error [41]. In subsequent RCTs, researchers are expected to not only ensure consistency in the inclusion of COPD patients but also standardize the duration, frequency, and movements of Qigong so as to guarantee the high quality of the original studies. After standardizing the movements of Qigong exercises, researchers can invite professionals to train the included patients so as to improve the standard of movements and the quality of the original research.

### 4.3. Strength and Limitations

This overview is the first to assess the current evidence for Qigong in the treatment of COPD from the perspectives of methodological quality, reporting quality, and evidence quality in all aspects, which can provide valuable information for clinicians' decision-making as well as suggestions for the future clinical trials with SRs/MAs. However, this overview also has some limitations, and we found that most of the included SRs/MAs were of poor quality, which may lead to the low credibility of the conclusions. Besides, this overview may be undesirably subjective at certain points. Although the assessments have been assessed and reviewed by two independent assessors, different assessors may have their own judgement on each factor, so results may vary.

## 5. Conclusions

The available evidence suggests that Qigong appears to be an effective and safe method of treating COPD. However, problems related to the methodology, evidence and reporting quality of SRs/MAs, and original clinical trials reduced the reliability of the results. To provide convincing evidence to researchers and clinicians in this field, methodological and reporting quality of SRs/MAs shall be further improved by conducting high-quality clinical studies of Qigong for COPD.

## Figures and Tables

**Figure 1:** The flowchart of the screening process.

**Table 1:** Search strategy for the PubMed database.

Query	Search term
#1	“Qigong” [Mesh]
#2	“Qi-gong” OR “Qi gong” OR “Chi chung” OR “Chi gong” OR “Chi Kung” OR “Qi Kung” OR “Jhi gong” OR “Chi gung” OR “Qi chung” OR “Ch'i kung” OR “Kung ch'i” OR Baduanjin OR Yijinjing OR Wuqinxi OR “Wu qin xi” OR “Shi'erduanjin” OR “changing tendon exercise” OR “five mimic-animal exercises” OR “six-character formula” OR “five elements balance work” OR “Longmen five elements skill” OR “Mawangdui” OR “Qigong”
#3	#1 OR #2
#4	Pulmonary Disease, Chronic Obstructive [Mesh]
#5	“Chronic Obstructive Lung Disease” OR “Chronic Obstructive Pulmonary Diseases” OR “COAD” OR “COPD” OR “Chronic Obstructive Airway Disease” OR “Chronic Obstructive Pulmonary Disease” OR “Airflow Obstruction, Chronic” OR “Airflow Obstructions, Chronic” OR “Chronic Airflow Obstructions” OR “Chronic Airflow Obstruction”
#6	#4 OR #5
#7	Meta-analysis as topic [mesh]
#8	“Systematic review” OR “meta-analysis” OR “meta analysis” OR “meta-analyses” OR “Review, Systematic” OR “Systematic reviews”
#9	#7 OR #8
#10	#3 AND #6 AND #9

**Table 2:** Characteristics of the included SRs/MAs.

Citation	Trials (subjects)	Intervention group	Control group	Quality assessment	Main results
Cao et al. [21]	31 (3,045)	Baduanjin+control group	CM, RA, BT	Cochrane criteria	Baduanjin exercise can improve lung function, exercise capacity, and quality of life in COPD patients.
Liu et al. [22]	20 (1,975)	Baduanjin+control group	CM, RA, BT	Physical therapy evidence database scale	Baduanjin exercise as a complementary therapy can improve exercise capacity, lung function, and quality of life in COPD patients.
Chen et al. [23]	12 (1,245)	Baduanjin+control group	CM, RA, BT	Cochrane criteria	Baduanjin exercise can improve lung function, improve exercise tolerance, and improve the quality of life of patients with COPD.
Han et al. [24]	9 (960)	Baduanjin+control group	CM, RA, BT	Cochrane criteria	Baduanjin exercise can improve lung function and exercise endurance in COPD patients.
Li et al. [25]	12 (1,179)	Baduanjin+control group	CM, RA, BT	Cochrane criteria	Baduanjin exercise can improve lung function and exercise endurance in COPD patients.
Xie et al. [26]	25 (2,058)	Baduanjin+control group	CM, RA, BT, HE	Cochrane criteria	Baduanjin exercise as a complementary therapy can improve exercise capacity, lung function, and quality of life in COPD patients.
Xiao et al. [27]	14 (920)	Liuzijue+control group	CM, RA, BT	Cochrane criteria	Liuzijue exercise can effectively improve dyspnea, exercise capacity, lung function, and quality of life in COPD patients.
Gao et al. [28]	16 (1,039)	Liuzijue+control group	CM, RA, BT	Cochrane criteria	Liuzijue exercise can effectively improve dyspnea, exercise capacity, lung function, and quality of life in COPD patients.
Liu et al. [29]	10 (578)	Liuzijue+control group	CM, RA, BT	Cochrane criteria	Liuzijue can improve exercise tolerance, respiratory function, and quality of life in patients with stable COPD.
Zhang et al. [30]	18 (1,036)	Liuzijue+control group	CM, RA, BT	Cochrane criteria	Liuzijue can improve exercise tolerance, respiratory function, and quality of life in patients with stable COPD.
Tong et al. [31]	10 (993)	Liuzijue, Baduanjin, Yijinjing, Wuqinxi+control group	CM, RA, BT	Cochrane criteria	Qigong exercise improved lung function, exercise capacity, and patients' quality of life within 6 months.
Li et al. [32]	20 (1,824)	Liuzijue, Baduanjin, Yijinjing+control group	CM, RA, BT	Cochrane criteria	Qigong exercise combined with basic therapy can improve lung function, exercise tolerance, and quality of life in stable COPD patients compared with basic therapy.
Yuan et al. [33]	8 (578)	Wuqinxi, Wuqinxi+control group	CM, RA, BT	Cochrane criteria	Wuqinxi exercise can improve lung function in COPD patients.

Note: CM: conventional medicine; RA: routine activities; BT: breathing training; HE: health education.

**Table 3:** Result of the AMSTAR-2 assessments.

Citation	Q1	Q2	Q3	Q4	Q5	Q6	Q7	Q8	Q9	Q10	Q11	Q12	Q13	Q14	Q15	Q16	Overall quality
Cao et al. [21]	Y	PY	Y	PY	Y	Y	N	Y	Y	N	Y	Y	Y	N	Y	Y	VL
Liu et al. [22]	Y	PY	Y	Y	Y	Y	N	Y	Y	N	Y	Y	Y	N	Y	Y	VL
Chen et al. [23]	Y	PY	Y	Y	Y	Y	N	Y	Y	N	Y	Y	Y	Y	Y	N	VL
Han et al. [24]	Y	PY	Y	Y	Y	Y	N	Y	Y	N	Y	Y	Y	N	N	Y	VL
Li et al. [25]	Y	PY	Y	Y	Y	Y	N	Y	Y	N	Y	Y	Y	Y	Y	N	VL
Xie et al. [26]	Y	PY	Y	Y	Y	Y	N	Y	Y	N	Y	Y	Y	Y	Y	Y	VL
Xiao et al., 2020 [27]	Y	Y	Y	PY	Y	Y	N	Y	Y	N	Y	Y	Y	N	N	Y	VL
Gao et al. [28]	Y	Y	Y	Y	N	Y	N	Y	Y	N	Y	Y	Y	Y	Y	Y	VL
Liu et al. [29]	Y	PY	Y	Y	Y	Y	N	Y	Y	N	Y	Y	N	Y	N	N	VL
Zhang et al. [30]	Y	PY	Y	PY	Y	Y	N	Y	Y	N	Y	Y	N	Y	N	Y	VL
Tong et al. [31]	Y	PY	Y	PY	Y	Y	Y	Y	Y	N	Y	Y	Y	Y	N	Y	VL
Li et al. [32]	Y	PY	Y	PY	Y	Y	N	Y	Y	N	Y	Y	Y	Y	N	Y	VL
Yuan et al. [33]	Y	PY	Y	PY	Y	Y	N	Y	Y	N	Y	Y	Y	Y	N	N	VL

Note: Y: yes; PY: partial yes; N: no; VL: very low; H: high; key areas are marked in red.

**Table 4:** Results of the PRISMA checklist.

Section/topic		Items	Cao et al. [21]	Liu et al. [22]	Chen et al. [23]	Han et al. [24]	Li et al. [25]	Xie et al. [26]	Xiao et al. [27]	Gao et al. [28]	Liu et al. [29]	Zhang et al. [30]	Tong et al. [31]	Li et al. [32]	Yuan et al. [33]	Number of yes or partially yes (%)
Title	Title	Item 1	Y	Y	Y	Y	Y	Y	Y	Y	Y	Y	Y	Y	Y	100%

Abstract	Abstract	Item 2	PY	PY	PY	PY	PY	PY	PY	PY	PY	PY	PY	PY	PY	100%

Introduction	Rationale	Item 3	Y	Y	Y	Y	Y	Y	Y	Y	Y	Y	Y	Y	Y	100%
	Objectives	Item 4	Y	Y	Y	Y	Y	Y	Y	Y	Y	Y	Y	Y	Y	100%

Methods	Eligibility criteria	Item 5	Y	Y	Y	Y	Y	Y	Y	Y	Y	Y	Y	Y	Y	100%
	Information sources	Item 6	Y	Y	Y	Y	Y	Y	Y	Y	Y	Y	Y	Y	Y	100%
	Search strategy	Item 7	Y	N	N	N	N	N	N	Y	N	N	Y	N	N	23.08%
	Selection process	Item 8	Y	Y	Y	Y	Y	Y	Y	N	Y	Y	Y	Y	Y	92.31%
	Data collection process	Item 9	Y	Y	Y	Y	Y	Y	Y	Y	Y	Y	Y	Y	Y	100%
	Data items	Item 10(a)	Y	Y	Y	Y	Y	Y	Y	Y	Y	Y	Y	Y	Y	100%
		Item 10(b)	Y	Y	Y	Y	Y	Y	Y	Y	Y	Y	Y	Y	Y	100%
	Study risk of bias assessment	Item 11	Y	Y	Y	Y	Y	Y	Y	Y	Y	Y	Y	Y	Y	100%
	Effect measures	Item 12	Y	Y	Y	Y	Y	Y	Y	Y	Y	Y	Y	Y	Y	100%
	Synthesis methods	Item 13(a)	Y	Y	Y	Y	Y	Y	Y	Y	Y	Y	Y	Y	Y	100%
		Item 13(b)	Y	Y	Y	Y	Y	Y	Y	Y	Y	Y	Y	Y	Y	100%
		Item 13(c)	Y	Y	Y	Y	Y	Y	Y	Y	Y	Y	Y	Y	Y	100%
		Item 13(d)	Y	Y	Y	Y	Y	Y	Y	Y	Y	Y	Y	Y	Y	100%
		Item 13(e)	N	N	Y	N	N	Y	N	Y	Y	N	N	Y	Y	46.15%
		Item 13(f)	N	N	N	N	N	N	N	Y	N	N	N	Y	Y	23.08%
	Reporting bias assessment	Item 14	Y	Y	Y	N	Y	N	N	Y	N	N	Y	N	N	46.15%
	Certainty assessment	Item 15	N	N	N	N	N	N	N	N	N	N	N	N	N	0%

Results	Study selection	Item 16(a)	Y	Y	Y	Y	Y	Y	Y	Y	Y	Y	Y	Y	Y	100%
		Item 16(b)	N	N	N	N	N	N	N	N	N	N	Y	N	N	7.69%
	Study characteristics	Item 17	Y	Y	Y	Y	Y	Y	Y	Y	Y	Y	Y	Y	Y	100%
	Risk of bias in studies	Item 18	Y	Y	Y	Y	Y	Y	Y	Y	Y	Y	Y	Y	Y	100%
	Results of individual studies	Item 19(a)	Y	Y	Y	Y	Y	Y	Y	Y	Y	Y	Y	Y	Y	100%
		Item 19(b)	Y	Y	Y	Y	Y	Y	Y	Y	Y	Y	Y	Y	Y	100%
	Results of syntheses	Item 20(a)	Y	Y	Y	Y	Y	Y	Y	Y	Y	Y	Y	Y	Y	100%
		Item 20(b)	Y	Y	Y	Y	Y	Y	Y	Y	Y	Y	Y	Y	Y	100%
		Item 20(c)	N	N	Y	N	Y	Y	N	Y	Y	Y	Y	Y	Y	69.23%
		Item 20(d)	N	N	Y	N	Y	Y	N	Y	N	Y	N	N	N	38.46%
	Reporting biases	Item 21	Y	Y	Y	N	Y	Y	N	Y	N	N	N	N	N	46.15%
	Certainty of evidence	Item 22	N	N	N	N	N	N	N	N	N	N	N	N	N	0%

Discussion	Discussion	Item 23(a)	Y	Y	Y	Y	Y	Y	Y	Y	Y	Y	Y	Y	Y	100%
		Item 23(b)	Y	Y	Y	Y	Y	Y	Y	Y	Y	Y	Y	Y	Y	100%
		Item 23(c)	Y	Y	Y	Y	Y	Y	Y	Y	Y	Y	Y	Y	Y	100%
		Item 23(d)	Y	Y	Y	Y	Y	Y	Y	Y	Y	Y	Y	Y	Y	100%

Other information	Registration and protocol	Item 24(a)	N	N	N	N	N	N	Y	Y	N	N	N	N	N	15.38%
		Item 24(b)	N	N	N	N	N	N	Y	Y	N	N	N	N	N	15.38%
		Item 24(c)	N	N	N	N	N	N	N	N	N	N	N	N	N	0%
	Support	Item 25	Y	Y	N	Y	N	Y	Y	Y	N	Y	Y	Y	N	69.23%
	Competing interests	Item 26	Y	Y	N	N	N	N	Y	Y	N	N	Y	N	N	38.46%
	Availability of data, code, and other materials	Item 27	Y	Y	Y	Y	Y	Y	Y	Y	Y	Y	Y	Y	Y	100%

Note: Y: yes; N: no; PY: partially yes.

**Table 5:** Results of evidence quality.

Citation	Outcomes	Limitations	Inconsistency	Indirectness	Imprecision	Publication bias	Quality
Cao et al. [21]	FEV1	-1①	-1②	0	0	-1④	Very low
	FVC	-1①	-1②	0	0	-1④	Very low
	FEV1/FVC	-1①	-1②	0	0	-1④	Very low
	6-MWD	-1①	-1②	0	0	-1④	Very low
	SGRQ	-1①	-1②	0	0	-1④	Very low
	CAT	-1①	-1②	0	0	-1④	Very low

Liu et al. [22]	6-MWD	0	-1②	0	0	0	Moderate
	FEV1	0	-1②	0	0	0	Moderate
	FEV1%	0	-1②	0	0	0	Moderate
	FVC	0	0	0	0	0	High
	FEV1/FVC	0	-1②	0	0	0	Moderate
	Quality of life	0	-1②	0	0	0	Moderate

Chen et al. [23]	FEV1	0	0	0	0	-1④	Moderate
	FEV1%	0	0	0	0	-1④	Moderate
	FVC	0	0	0	0	-1④	Moderate
	FEV1/FVC	0	-1②	0	0	-1④	Low
	CAT	0	-1②	0	0	-1④	Low

Han et al. [24]	6-MWD	0	0	0	-1③	-1④	Low
	FEV1	0	-1②	0	0	-1④	Low
	FEV1%	0	0	0	0	-1④	Moderate
	FVC	0	0	0	-1③	-1④	Low
	FEV1/FVC	0	-1②	0	-1③	-1④	Very low

Li et al. [25]	FEV1/pred%	0	-1②	0	0	-1④	Low
	FEV1	0	-1②	0	-1③	0	Low
	FEV1%	0	-1②	0	0	0	Moderate
	FVC	0	0	0	-1③	0	Moderate
	6-MWD	0	-1②	0	0	0	Very low

Xie et al. [26]	6-MWD	-1①	-1②	0	0	-1④	Very low
	FEV1	-1①	-1②	0	0	-1④	Very low
	FEV1%	-1①	-1②	0	0	0	Low
	FVC	-1①	-1②	0	0	-1④	Very low
	FEV1/FVC	-1①	-1②	0	0	-1④	Very low
	CAT	0	-1②	0	-1③	-1④	Very low
	SGRQ	-1①	-1②	0	0	-1④	Very low
	WHOQOL-BREF	0	-1②	0	0	-1④	Low

Xiao et al. [27]	MRC	0	-1②	0	-1③	-1④	Very low
	6-MWD	0	0	0	-1③	-1④	Low
	FEV1	0	-1②	0	0	-1④	Low
	FEV1/pred%	-1①	-1②	0	0	-1④	Very low
	FEV1/FVC	0	-1②	0	0	-1④	Low
	CAT	0	-1②	0	0	-1④	Low
	SGRQ	0	-1②	0	-1③	-1④	Very low

Gao et al. [28]	MRC	0	0	0	0	-1④	Moderate
	6-MWD	0	0	0	0	0	High
	FEV1	0	0	0	0	0	High
	FEV1%	0	-1②	0	0	0	Moderate
	FEV1/FVC	0	-1②	0	0	0	Moderate
	Quality of life	0	-1②	0	0	-1④	Low

Liu et al. [29]	6-MWD	-1①	0	0	-1③	-1④	Very low
	FEV1	-1①	0	0	-1③	-1④	Very low
	FEV1%	-1①	0	0	-1③	-1④	Very low

Zhang et al. [30]	MRC	-1①	0	0	-1③	-1④	Very low
	6-MWD	0	-1②	0	0	-1④	Low
	FEV1	-1①	-1②	0	-1③	-1④	Very low
	FEV1%	-1①	-1②	0	0	-1④	Very low
	CAT	-1①	0	0	-1③	-1④	Very low

Tong et al. [31]	6-MWD	0	-1②	0	0	-1④	Low
	FEV1	0	-1②	0	0	-1④	Low
	FEV1/FVC	0	0	0	0	-1④	Moderate
	FEV1%	0	-1②	0	0	-1④	Low
	CAT	0	-1②	0	-1③	-1④	Very low

Li et al. [32]	FEV1% (3 months)	0	0	0	0	-1④	Moderate
	FEV1% (6 months)	0	-1②	0	0	-1④	Low
	FEV1/FVC (3 months)	0	-1②	0	0	-1④	Low
	FEV1/FVC (6 months)	0	-1②	0	0	-1④	Low
	CAT	0	0	0	-1③	-1④	Low
	6-MWD (3 months)	0	0	0	0	-1④	Moderate
	6-MWD (6 months)	0	-1②	0	0	-1④	Low

Yuan et al. [33]	FEV1	-1①	-1②	0	-1③	-1④	Very low
	FEV1%	-1①	-1②	0	-1③	-1④	Very low
	FEV1/FVC	-1①	-1②	0	0	-1④	Very low
	FEV1/pred%	-1①	-1②	0	-1③	-1④	Very low
	6-MWD	-1①	-1②	0	-1③	-1④	Very low

Note: ① the included studies have a large bias in methodology such as randomization, allocation concealment, and blinding. ② The confidence interval overlaps less or the *I*^2^ value of the combined results was larger. ③ The sample size from the included studies does not meet the optimal sample size or the 95% confidence interval crosses the invalid line. ④ The funnel chart is asymmetry; FEV1: the forced expiratory volume in one second; FVC: forced vital capacity; 6-MWD: 6 min walking distance; FEV1/FVC: the amount of air exhaled in the first second divided by all of the air exhaled during a maximal exhalation; SGRQ: St George's respiratory questionnaire; CAT: COPD assessment test; FEV1%: percentage of the forced expiratory volume in one second; QOL: quality of life; WHOQOL-BREF: the World Health Organization on quality of life brief scale; MRC: medical research council dyspnea scale; FEV1%pred: the percentage of predicted values of FEV1.

**Table 6:** Summary of evidence.

Citation	Outcomes	Studies (participants)	Heterogeneity	Relative effect (95% CI)	*P* value
Cao et al. [21]	FEV1	17 (1,395)	83%	MD = 0.23 (0.15, 0.31)	*P* < 0.00001
	FVC	13 (1,033)	61%	MD = 0.19 (0.08, 0.30)	*P* = 0.0007
	FEV1/FVC	20 (1,808)	74%	MD = 3.85 (2.19, 5.51)	*P* < 0.00001
	6-MWD	18 (1,562)	96%	MD = 43.83 (29.47, 58.20)	*P* < 0.00001
	SGRQ	4 (280)	54%	MD = −7.71 (−10.54, −4.89)	*P* < 0.00001
	CAT	7 (802)	78%	MD = −2.56 (−4.13, −1.00)	*P* = 0.001

Liu et al. [22]	6-MWD	10 (1,160)	66%	Hedge′s *g* = 0.69 (0.44, 0.94)	*P* < 0.001
	FEV1	10 (809)	68%	Hedge′s *g* = 0.47 (0.22, 0.73)	*P* < 0.001
	FEV1%	13 (1,417)	54%	Hedge′s *g* = 0.38 (0.21, 0.56)	*P* < 0.001
	FVC	8 (674)	14%	Hedge′s *g* = 0.39 (0.22, 0.56)	*P* < 0.001
	FEV1/FVC	13 (1,284)	53%	Hedge′s *g* = 0.5 (0.33, 0.68)	*P* < 0.001
	Quality of life	7 (746)	77%	Hedge′s *g* = −0.45 (-0.77, -0.12)	*P* < 0.05

Chen et al. [23]	FEV1	7 (525)	0%	MD = 0.25 (0.12, 0.38)	*P* < 0.001
	FEV1%	10 (1,005)	26%	MD = 6.71 (4.25, 9.18)	*P* < 0.001
	FVC	6 (423)	42%	MD = 0.16 (0.01, 0.31)	*P* = 0.04
	FEV1/FVC	9 (925)	71%	MD = 4.90 (2.43, 7.38)	*P* < 0.001
	CAT	5 (679)	78%	MD = −1.84 (-3.50, -0.19)	*P* < 0.05

Han et al. [24]	6-MWD	4 (346)	28%	MD = 45.27 (40.11, 50.42)	*P* < 0.01
	FEV1	5 (450)	82%	MD = 0.26 (0.14, 0.37)	*P* < 0.01
	FEV1%	7 (775)	36%	MD = 6.02 (5.02, 7.01)	*P* < 0.01
	FVC	3 (266)	0%	MD = 0.27 (0.06, 0.48)	*P* = 0.01
	FEV1/FVC	6 (423)	85%	MD = 3.63 (-0.18, 7.43)	*P* = 0.06

Li et al. [25]	FEV1/pred%	9 (985)	67%	MD = 6.86 (4.13, 9.60)	*P* < 0.01
	FEV1	4 (346)	75%	MD = 0.30 (0.14, 0.46)	*P* < 0.01
	FEV1%	8 (905)	73%	MD = 4.50 (1.84, 7.16)	*P* < 0.01
	FVC	3 (246)	0%	MD = 0.34 (0.13, 0.54)	*P* < 0.01
	6-MWD	6 (476)	92%	MD = 56.35 (37.55, 75.16)	*P* < 0.01

Xie et al. [26]	6-MWD	12 (895)	83%	SMD = 1.33 (0.97, 1.68)	*P* < 0.001
	FEV1	12 (895)	94%	SMD = 1.05 (0.56, 1.55)	*P* < 0.001
	FEV1%	15 (1,848)	86%	SMD = 0.50 (0.24, 0.76)	*P* = 0.0002
	FVC	9 (925)	68%	SMD = 0.26 (0.03, 0.50)	*P* = 0.03
	FEV1/FVC	14 (1,762)	83%	SMD = 0.44 (0.20, 0.68)	*P* = 0.0004
	CAT	3 (443)	87%	SMD = −0.56 (-1.24, 0.12)	*P* = 0.11
	SGRQ	3 (762)	81%	SMD = −1.36 (-1.74,-0.98)	*P* < 0.001
	WHOQOL-BREF	2 (852)	73%	SMD = 0.94 (0.66, 1.22)	*P* < 0.001

Xiao et al. [27]	MRC	3 (136)	62%	MD = −0.73 (-1.13, -0.33)	*P* < 0.05
	6-MWD	6 (274)	0%	MD = 17.78 (7.97, 27.58)	*P* < 0.05
	FEV1	8 (502)	83%	MD = 0.23 (0.07, 0.38)	*P* < 0.05
	FEV1/pred%	10 (580)	97%	MD = 7.59 (2.92, 12.26)	*P* < 0.05
	FEV1/FVC	12 (769)	95%	MD = 6.81 (3.22, 10.40)	*P* < 0.05
	CAT	4 (341)	56%	MD = −2.29 (-3.27, -1.30)	*P* < 0.05
	SGRQ	5 (297)	63%	MD = −9.85 (-13.13, -6.56)	*P* < 0.05

Gao et al. [28]	MRC	3 (459)	42%	MD = −0.73 (-0.96, -0.50)	*P* < 0.001
	6-MWD	9 (805)	43%	MD = 21.89 (14.67, 29.11)	*P* < 0.001
	FEV1	9 (560)	5%	MD = 0.19 (0.13, 0.24)	*P* < 0.001
	FEV1%	13 (861)	57%	MD = 7.14 (6.09, 8.18)	*P* < 0.001
	FEV1/FVC	13 (890)	83%	MD = 4.2 (3.26, 5.14)	*P* < 0.001
	Quality of life	7 (780)	56%	SMD = −0.84 (-1.12, -0.55)	*P* < 0.001

Liu et al. [29]	6-MWD	5 (326)	0%	MD = 22.62 (10.49, 34.75)	*P* < 0.05
	FEV1	5 (247)	0%	MD = 0.10 (0.01, 0.18)	*P* < 0.05
	FEV1%	5 (247)	24%	MD = 3.08 (0.18, 5.97)	*P* = 0.04

Zhang et al. [30]	MRC	5 (228)	22%	MD = −0.55 (-0.75, -0.36)	*P* < 0.001
	6-MWD	9 (475)	74%	MD = 33.76 (18.99, 48.52)	*P* < 0.001
	FEV1	6 (337)	67%	MD = 0.19 (0.06, 0.31)	*P* = 0.01
	FEV1%	13 (644)	89%	MD = 6.08 (2.55, 9.62)	*P* = 0.0007
	CAT	4 (266)	4%	MD = −2.69 (-3.34, -2.03)	*P* < 0.001

Tong et al. [31]	6-MWD	8 (629)	90%	MD = 30.57 (19.61, 41.53)	*P* < 0.001
	FEV1	5 (449)	90%	MD = 0.32 (0.09, 0.56)	*P* < 0.001
	FEV1/FVC	6 (535)	47%	MD = 2.66 (1.32, 2.26)	*P* < 0.001
	FEV1%	5 (455)	61%	MD = 6.04 (2.58, 9.5)	*P* = 0.006
	CAT	3 (258)	84%	MD = −5.54 (-9.49, -1.59)	*P* = 0.002

Li et al. [32]	FEV1% (3 months)	10 (695)	36%	MD = 5.34 (2.70, 7.98)	*P* < 0.001
	FEV1% (6 months)	9 (1,006)	86%	MD = 5.35 (2.58, 8.12)	*P* = 0.0001
	FEV1/FVC (3 months)	10 (695)	66%	MD = 4.49 (1.66, 7.31)	*P* = 0.002
	FEV1/FVC (6 months)	11 (926)	79%	MD = 2.53 (0.38, 4.68)	*P* = 0.02
	CAT	5 (262)	6%	MD = −4.18 (-5.52, -2.84)	*P* < 0.001
	6-MWD (3 months)	6 (480)	45%	MD = 22.10 (12.43, 31.78)	*P* < 0.001
	6-MWD (6 months)	9 (628)	95%	MD = 44.46 (20.59, 68.34)	*P* < 0.001

Yuan et al. [33]	FEV1	4 (258)	73%	MD = 0.39 (0.21, 0.57)	*P* < 0.001
	FEV1%	4 (273)	97%	MD = 4.41 (-1.97, 10.79)	*P* = 0.18
	FEV1/FVC	8 (577)	97%	MD = 10.39 (5.44, 15.35)	*P* < 0.001
	FEV1/pred%	4 (324)	95%	MD = 8.44 (0.40, 16.48)	*P* = 0.04
	6-MWD	4 (278)	93%	MD = 63.42 (34.06, 92.79)	*P* < 0.001

Note: SMD: standardized mean difference; MD: mean difference; FEV1: forced expiratory volume in one second; FVC: forced vital capacity; 6-MWD: 6 min walking distance; FEV1/FVC: the amount of air exhaled in the first second divided by all of the air exhaled during a maximal exhalation; SGRQ: St George's respiratory questionnaire; CAT: COPD assessment test; FEV1%: percentage of the forced expiratory volume in one second; QOL: quality of life; WHOQOL-BREF: the World Health Organization on quality of life brief scale; MRC: medical research council dyspnea scale; FEV1%pred: the percentage of predicted values of FEV1.

## Data Availability

The datasets analyzed during the current study are available from the corresponding author on reasonable request.
